# Analysis of Center of Pressure Signals by Using Decision Tree and Empirical Mode Decomposition to Predict Falls among Older Adults

**DOI:** 10.1155/2021/6252445

**Published:** 2021-11-25

**Authors:** Fang-Yin Liao, Chun-Chang Wu, Yi-Chun Wei, Li-Wei Chou, Kang-Ming Chang

**Affiliations:** ^1^Department of Physical Medicine and Rehabilitation, China Medical University Hospital, 40402 Taichung, Taiwan; ^2^Department of Traditional Chinese Medicine, Asia University Hospital, 41354 Taichung, Taiwan; ^3^School of Chinese Medicine, College of Chinese Medicine, China Medical University, 40402 Taichung, Taiwan; ^4^Department of Computer Science and Information Engineering, Asia University, 41354 Taichung, Taiwan; ^5^Department of Physical Medicine and Rehabilitation, Asia University Hospital, Asia University, 41354 Taichung, Taiwan; ^6^Department of Physical Therapy and Graduate Institute of Rehabilitation Science, China Medical University, 40402 Taichung, Taiwan; ^7^Department of Medical Research, China Medical University Hospital, China Medical University, 40402 Taichung, Taiwan; ^8^Department of Digital Media Design, Asia University, 41354 Taichung, Taiwan

## Abstract

Falls put older adults at great risk and are related to the body's sense of balance. This study investigated how to detect the possibility of high fall risk subjects among older adults. The original signal is based on center of pressure (COP) measured using a force plate. The falling group includes 29 subjects who had a history of falls in the year preceding this study or had received high scores on the Short Falls Efficacy Scale (FES). The nonfalling group includes 47 enrollees with no history of falls and who had received low scores on the Short FES. The COP in both the anterior–posterior and mediolateral direction were calculated and analyzed through empirical mode decomposition (EMD) up to six levels. The following five features were extracted and imported to a decision tree algorithm: root-mean-square deviation, median frequency, total frequency power, approximate entropy, and sample entropy. The results showed that there were a larger number of statistically different feature parameters, and a higher classification of accuracy was obtained. With the aid of empirical mode decomposition, the average classification accuracy increased 10% and achieved a level of 99.74% in the training group and 96.77% in the testing group, respectively.

## 1. Introduction

With the advent of our aging society, many topics related to the health of the elderly have attracted more and more attention year after year, especially the concept of preventive medicine. The most relevant things to the healthy development of the elderly are falls, body balance, and daily activity. Falling is the second leading cause of accidental death after road injuries Therefore, fall detection is an important research topic. The decline of overall balance ability is one of the important indicators of the aging process of body function and also one of the factors that causes the fall. Testing the balance of the elderly can be used to assess the risk of falls. At present, detecting falls can be divided into two categories: prediction and immediate fall detection. Fall detection is currently dominated by wearable devices [1] or by infrared sensing [2]. Wearable fall detection systems mainly use accelerometers for sensing, which are placed on different parts of the human body and can distinguish activities of daily living. Although wearable devices are conducive to detecting real-time falls, aging is a gradual process of change; before a fall, the elderly are usually reluctant to wear a fall detector. It is beneficial to provide a method to detect the risk assessment for the elderly. They will have higher will to use wearable device if they are notified with high falling risk.

One of the physiological signals used in the study of the balance mechanism in the human body is the center of pressure (COP), which is measured by using a biomechanical force plate in which the parallel force changes with the body's sense of balance [3, 4]. The force plate measures forces and torques on three axes: forward–backward, left–right, and up–down. Several studies have used COP data to assess the body's sense of balance and falls [5, 6]. For example, Santos et al. measured the COP of 163 enrollees who stood still for 60 s under four measurement conditions: eyes open on a rigid surface, eyes closed on a rigid surface, eyes open on a foam mat, and eyes closed on a foam mat [7]. Measurements under each condition were performed three times for each enrollee in a randomized order. The enrollees consisted of young adults, older adults with a history of falls in the year prior, and older adults with no history of falls in the year prior. In addition to measuring COP time series signals under four conditions, Santos et al. measured the enrollees' personal and health conditions (e.g., age, height, weight, BMI, and diseases) by administering questionnaires related to falls and physical activity (i.e., International Physical Activity Questionnaire, Falls Efficacy Scale FES, Mini Balance Evaluation Systems Test, Trail Making Tests A and B, and F12M). F12M queried the enrollees about the number of falls they had in the 12 months prior. With the same data, Montesinos et al. continued the study by calculating the COP using nonlinear parameters (i.e., approximate entropy and sample entropy). In addition, they discussed the effects of changing input parameters *m*, *r*, and N (data length of 30 and 60 s) on approximate entropy and sample entropy values in the COP time series [8]; the study revealed that more significant differences between young and older adults were observed in the nonlinear parameters compared with the linear COP parameters. There were no observed significant differences between older adults who had not experienced falls in the 12 months prior and those who had experienced falls in the last 12 months (i.e., nonfallers and fallers) across all of the parameters. Nonlinear parameters are often used for the characteristic extraction of physiological signals and achieve well-founded performance [9, 10]. Chang further investigated the topic by analyzing COP signals using empirical mode decomposition (EMD) and extracting intrinsic mode functions (IMFs) to compute the entropy features. Chang discovered significant differences between nonfallers and fallers in multiple parameters [11].

The EMD algorithm decomposes data into IMFs for analysis and is particularly useful for processing nonlinear and nonsteady signals. Similar to filter banks, EMD gradually computes IMFs by repeating a screening procedure. The initially computed IMFs contain the highest frequency components. Then, signals of different frequency components are gradually decomposed until becoming sine waves, as if passing through bandpass filters [12]. Unlike bandpass filters with a fixed bandwidth, the IMF components decomposed through EMD vary with the features of the input signals. That is, the EMD algorithm follows a concept similar to that of dynamic bandwidth filters. Several studies have applied EMD to identify meaningful signal components in the processing of physiological signals, such as in electrocardiograms [13], electroencephalograms [14], and fetal heart sound [15]. Compared with the conventional method, in which features are directly extracted from original signals, decomposing IMFs through EMD and then extracting features from the decomposed IMFs is a more effective method for identifying differences between extracted features. This method considerably improves the subsequent signal classification performance.

The combination of physiological signals and artificial intelligence algorithms has become prevalent in clinical classification and diagnosis in recent years. Machine learning is an effective tool for classification [16]. Studies on fall risk predictors have discovered that, by using machine learning to create effective classification models, multiple functions and nonlinear algorithms can be used to classify fall risks [17]. The majority of studies have used dynamic motion analysis to predict the risk of falls in older adults [18, 19]. The decision tree algorithm is a notable algorithm with explainable reasoning [20, 21]. Decision trees are a nonparametric supervised learning method used for classification and regression. By creating a model that predicts the value of the target variable through learning, decision rules can be determined by data features. A decision tree can identify each stage of decision-making by organizing the multiple decision points.

The automatic identification system for COP detection of falls has not yet been published. The objective of this study was to develop an autonomic algorithm to detect the possibility of high fall risk subjects among older adults, with the time domain, frequency domain, and nonlinear domain COP feature derived from EMD. In addition, this study used the decision tree algorithm to classify enrollees into the fall and nonfall groups. Finally, an investigation was made into the differences between the fall and nonfall groups in terms of COP measured under four conditions, a subject that studies have rarely explored.

## 2. Materials and Methods

### 2.1. COP Data

This study used test data collected by Santos and Duarte who stood still for 60 s on a force platform (OPT400600-1000; AMTI, Watertown, MA, USA) under four different conditions [7]. Measurements under the four conditions were performed three times for each enrollee in a randomized order. The four conditions were defined as follows: on a rigid surface with eyes closed (CR); on a rigid surface with eyes open (OR); on a foam mat with eyes closed (CF); and on a foam mat with eyes open (OF). *C*4 = CR + OR + CF + OF is the combination of four measurement conditions. COP measurements were performed at a sampling frequency of 100 Hz; the outputs of the force plate were force (*Fx*, *Fy*, *Fz*) and moment (*Mx*, *My*, *Mz*) data. The enrollees, aged >65 years, were divided into the fall and nonfall groups on the basis of their history of falls in the 12 months prior and their responses to the FES-International questionnaire. The 47 enrollees who had not experienced falls in the 12 months prior were allocated to the nonfall group, and the 29 enrollees who had fallen once or twice in the 12 months prior or had received high scores on the Short FES were allocated to the fall group.  Table 1 summarizes the demographic data of the two groups of enrollees. COP signals in the anterior–posterior (COP*x*) and mediolateral (COP*y*) directions were calculated for subsequent feature extraction.

### 2.2. EMD Formula

EMD of signal *x*(*t*) is described as follows [22]:

Step 1: Set the maxima and minima of *x*(*t*).
Step 2: The maxima and minima are connected to form the upper and lower envelopes.
Step 3: Compute *m*(*t*), the mean function of the upper and lower envelopes.
    Step 4: Solve *d*(*t*) = *x*(*t*) − *m*(*t*).
    Step 5: If *d*(*t*) is the zero-mean process, the computation ends, and *d*(*t*) becomes the first IMF (IMF1). Otherwise, replace *x*(*t*) with *d*(*t*), and return to Step 1.
    Step 6: Residual signal *r*(*t*) = *x*(*t*) − IMF1(*t*).
    Step 7: Replace *x*(*t*) with *r*(*t*) and repeat Steps 1 to 6 to compute the second IMF, IMF2(*t*). After *n* iterations, IMFn(*t*) is obtained. The computation does not stop until *r*(*t*) becomes a monotonic function.

The original data are decomposed into *n* IMFs, IMF(*t*), and a residual signal *r*(*t*).

The programs used in this study are written in *R* language. To perform EMD, an EMD package was downloaded, library(EMD) was loaded, the command “emd” was used, and IMF1–IMF7 were extracted. Because IMF7 consists of signals decomposed into sine waves with no information related to COP, decomposition was performed to only the 6th level (IMF6).  Figure 1 presents the process of decomposition of one original COP*x* signal from the fall and nonfall groups to IMF1–IMF6.

### 2.3. COP Features

The two signal sources, COPx and COPy, were decomposed into IMF1–IMF6 through EMD. Then, five feature parameters for the time series signal were computed, namely, root-mean-square deviation (RMSD), representing the time domain feature parameter; median frequency and total frequency power, representing the frequency domain feature parameters; and approximate entropy and sample entropy, representing the nonlinear parameters. The computation of approximate entropy and sample entropy required the use of commands “approx_entropy” and “sample_entropy,” respectively, in the R-language pracma package. Entropy had two input parameters, namely, dimension = 2 and *r* = 0.2 × STD, where STD denotes the standard deviation of the input signal. In the command “sample_entropy, tau = 1.” The frequency spectrum was computed by using the command “pspectrum” in the *R*-language psd package. The coding rules for the feature parameters were divided into three levels: level 1 represents signal source, COPx, or COPy; level 2 represents the corresponding IMF function level; and level 3 represents the five features.  Table 2 presents the feature parameters and their code numbers. For example, x.0.1 corresponds to the RMSD parameter computed from the original COP*x* signal, and *y*.2.4 corresponds to the approximate entropy parameter computed from COPy to the second IMF.

### 2.4. DT Classification and Evaluation

The five feature parameters computed in Section 2.3 were further divided into five measurement conditions: CF, OF, CR, OR, and *C*4 (the four conditions combined). The COP*x* and COP*y* signals were decomposed from the original signals into IMF1–IMF6 as input parameters. The R-language command “CART” was used to perform decision tree classification, and the training–testing data ratio was kept as 80 : 20. The enrollees were classified into the fall and nonfall groups, and the results of the classification were divided into one of the four following categories based on a comparison with the enrollees' history of falls: older adults who were classified by the decision tree into the fall group and had a history of falls (TP); older adults who were classified by the decision tree into the fall group but had no history of falls (FP); older adults who were classified by the decision tree into the nonfall group but had history of falls (FN); older adults who were classified by the decision tree into the nonfall group and had no history of falls (TN).

The following three categorical parameters are defined in terms of TP, FP, FN, and TN:

(1) $$\begin{array}{c} \text{Accuracy}=\left(\frac{\left(\text{TP}+\text{TN}\right)}{\left(\text{TP}+\text{FN}+\text{TN}+\text{FP}\right)}*100\right),\\ \text{Specificity}=\left(\frac{\text{TN}}{\left(\text{TN}+\text{FP}\right)}*100\right),\\ \text{Sensitivity}=\left(\frac{\text{TP}}{\left(\text{TP}+\text{FN}\right)}*100\right). \end{array}$$

The decision tree classification was repeated 20 times under the same conditions to compute the mean and standard deviation for the accuracy, specificity, and sensitivity of the classification into training and testing groups.

### 2.5. Statistics

The following hypotheses were proposed:

  H1: EMD can produce more statistically different parameters.
  H2: Parameters derived from EMD can improve the accuracy of enrollee classification.
  H3: Statistically different feature parameters vary among methods of COP measurement and their combinations.
  H4: The methods of COP measurement and their combinations affect the accuracy of enrollee classification

All data is processed with following statistics:

#### 2.5.1. Descriptive Statistics

This study divided the feature parameters of the enrollees' data into the fall and nonfall groups to compute the mean and standard deviation of the feature parameters for each group. After the decision tree classification, the mean and standard deviation of the accuracy, sensitivity, and specificity in the training and testing groups were calculated for 20 rounds of classification.

#### 2.5.2. *T*-Test

The input COP parameters of fall and nonfall were computed for *t*-test, with a significance level of *α* = 0.05.  Figure 2 presents the experimental process, and Appendix A presents the codes used in this study.

## 3. Results

### 3.1. COP Feature Distribution between Two Groups

Table 3 demonstrates the feature distribution with C4 measurement condition. The detailed feature distribution of each subject among four data measurement conditions and combined measurement condition is listed in Appendix A, inclusive of mean and standard derivation of both fall and nonfall groups. The statistical differences between the fall and nonfall groups under the four measurement conditions were also evaluated, as shown in Appendix A. The thorough statistically different features are listed in Table 4.  Table 5 lists the numbers of statistically significant features on different COP measurement conditions derived from Table 3. From Table 4, there were 32 EMD-derived features and three original signals (*y*.0.4, *x*.0.5, and *y*.0.5) from *C*4 signals; eleven EMD-derived features were from OF signals; three EMD-derived features and one original signal (*y*.0.5) were from CF signals; fifteen EMD-derived features and two original signals (*x*.0.5 and *y*.0.5) were from CR signals; 25 EMD-derived features and two original signals (*x*.0.5 and *y*.0.5) were from OR signals.

### 3.2. Finding for COP Feature Distribution among Different Data Recording Conditions

According to the results derived from Tables 4 and 5, there are several findings with different data recording conditions.

#### 3.2.1. Eyes Open versus Eyes Closed

In terms of the number of statistically different parameters, OR > CR and OF > CF, maintaining balance with the eyes closed was more difficult for the fall group. The degree of body sway was greater in the fall group than in the nonfall group, causing the intergroup gap to increase. Maintaining a balance with the eyes open was relatively easy.

#### 3.2.2. Rigid Standing Surface versus Foam Mat Standing Surface

In terms of the number of statistically different parameters, OR > OF and CR > CF, the results showed that because the rigid surface was relatively stable and the foam mat was relatively unstable, the nonfall group had difficulties maintaining stability on the foam mat. Because of this result, the differences between the fall and nonfall groups were reduced on the foam mat surface.

#### 3.2.3. *C*4 Data Recording Conditions versus Separate Data Recording Condition

A total of 35 statistically different parameters were derived from *C*4 (four conditions combined). A comparison of the data in Table 4 revealed the following 11 parameters observed in the individual condition measurements but not in *C*4 condition: *x*.2.3, *x*.3.1, *x*.3.3, *x*.4.1, *x*.4.3, *x*.5.1, *x*.5.3, *x*.6.1, *x*.6.3, *y*.1.4, *y*.3.4. The following seven parameters were not observed in the individual condition measurements but were observed in C4: *x*.1.2, *x*.2.5, *y*.4.4, *y*.4.5, *y*.6.4, *y*.6.5. These results indicated that although *C*4 represents the combination of the four measurement conditions (i.e., CR, CR, OR, and OF), several features observed in *C*4 were different from those observed in the individual condition measurements. This phenomenon suggests that COP signals should be measured under all four conditions. These three findings support H3: statistically different feature parameters vary among methods of COP measurement and their combinations. The feature parameters derived from each COP measurement condition affected the difference in the statistics between the fall and nonfall groups.

### 3.3. Finding for COP Features with EMD Processing

In terms of the number of statistically different parameters, *C*4 yielded 32 IMF-derived features and only three raw signals. As a result, the parameters derived from EMD significantly increased the number of statistically different parameters. IMF5 resulted in the largest number of statistically different parameters. This finding supports H1: EMD can produce a larger number of statistically different parameters. The feature parameters were input into the decision tree for classification, which divided them into the fall and nonfall groups.

At the end of Table 5, *C*4 yielded three time-domain derived features, 10 frequency-domain derived features, and also 22 nonlinear-domain derived features. Nonlinear domain features contributed more statistically different features than frequency domain and time-domain features.

### 3.4. Decision Tree Classification Result between Fall and Nonfall Groups

The classifier performed 20 rounds of classification to obtain the mean and standard deviation of classifier performance. The detailed classification performance with single feature and ten features set of raw COP and IMF under four data measurement conditions are listed in Appendix B.  Figure 3 is the classifier accuracy of testing group. According to Figure 3, the use of 10 original feature parameters for time domain, frequency domain, and nonlinear domain to classify the *C*4 input data yielded a testing group classification accuracy of 84.09% (with standard derivation of 4.61%). The use of 10 feature parameters derived from EMD1 to EMD6 yielded testing group classification accuracies of 88.13% (4.39%), 91.10% (5.84%), 92.34% (5.21%), 88.22% (8.12%), 95.76% (5.43%), and 96.77% (3.85%), respectively. This result supports H2 because the EMD-derived features improved classification accuracy (H2: parameters derived from EMD can improve the enrollee classification accuracy). The other finding from Figure 3 is that the classification accuracy of *C*4 is greater than the individual data recording condition, either by using 10 original feature parameters or those yielded by using EMD1 to EMD6. This finding supports H4: methods of COP measurement and their combinations affect the accuracy of enrollee classification.

## 4. Discussion

There are several interesting findings. First, this article is the first paper to use COP signals and AI to classify fall and nonfall elderly. The reason for the difficulty of this topic is to first find the COP feature with statistical differences. Feature parameters have rarely been yielded in studies on the application of COP feature parameters to distinguish fall and nonfall groups. Montesinos et al. [8] discovered that significant differences in approximate entropy were only observed for certain combinations of *m*, *r*, and *N*. These results are consistent with those of this study. For example, *y*.0.4, *x*.0.5, and *y*.0.5 were statistically different feature parameters derived from *C*4. The present study differed from that of Montesinos et al. in that both the enrollees who had experienced falls in the 12 months prior (as indicated by the self-reported F12M) and the enrollees who had not experienced falls in the 12 months prior but received high scores on the FES were allocated to the fall group. This difference might have caused slight differences in the results. However, both studies noted that statistically different feature parameters for the COP of older adults between fall and nonfall groups were lacking.

The second finding is that the features derived from the combination of four COP recording conditions, and being processed by EMD, increases the number of parameters with statistical differences between fall and nonfall groups, in which nonlinear parameters are the majority. After the COP signal is decomposed by EMD, the testing group classification accuracy can be increased by 10% in IMF5 and IMF6 to 95%-96%, compared with corresponding raw COP derived features. The fact that EMD can extract a larger number of feature parameters to distinguish fall and nonfall groups than can the original signals without EMD may be attributable to the characteristics of EMD. The initially computed IMFs derived from EMD contain the highest frequency components, and the frequency decreases with each level of decomposition. EMD resembles a continuous-time bandpass filter bank with nonfixed bandwidths. The IMF number is inversely proportional to the frequency. Signals of different frequency components are gradually decomposed until becoming sine waves. The components of the COP signals were likely the same for the fall and nonfall groups with only a few differences that can be identified by using the characteristics of the EMD analysis method. A group of nearly identical signals may only differ in certain frequency bands, and the performance of EMD can highlight the different signal components and thus produce statistical differences. In terms of COP*x*, the different parameters were mainly observed in IMF1–IMF4, which was the midband of the signal. The different parameters of the COP*y* were distributed among IMF2–IMF5 and were nonlinear. EMD can separate the COP components related to falls.

The COP data used in this study were measured under four conditions, namely, CF, OF, CR, and OR. This study proposed an innovative method in terms of the necessity of the four measurement conditions. The feature parameters of COP measured under the four conditions differed between the fall and nonfall groups. According to Tables 4 and 5, new feature parameters that were not observed in combination of the original four measurements, CF, OF, CR, OR, were observed in *C*4. Therefore, measuring COP under four conditions and combining the results can increase the yield of new statistically different parameters.

There are several limitations of this study. First, the sample size of the experiment is small. The data is taken from a public database, with only 29 falling elderly people and the control group of 47 elderly people. Although this subject size is sufficient to examine the decision classification performance, it is expected to check the classifier performance with more subjects, especially coming from different countries.

Second, only 10COP parameters were used this time. The linear and nonlinear parameters were included, of which the linear parameters were low in computation, but the nonlinear parameters could provide a large number of parameters with statistical differences. The third limitation is the classification algorithm. This article applies only decision tree analysis for classification. There are many supervised classification algorithms, such as neuronetwork [23], support vector machine [24], and deep leaning [25]. Therefore, a broader study of the effects of other nonlinear parameters applied to COP, as well as comparing different classifiers, is an interesting topic in the future study.

## 5. Conclusions

This study uses COP data to detect elderly people with a history of falls. This is combined with four COP measurement criteria: eyes closed/open and standing on rigid/foam mat surface, and followed with EMD processing, COP signals produced a larger number of statistically different parameters. The decomposed parameters can improve the accuracy of fall and nonfall classification. The 6th level of IMF (IMF6) achieved the highest classification accuracy; the average accuracy of the corresponding training group 99.74%, and the average testing group accuracy is 96.77%. Thus, a larger number of statistically different feature parameters and a higher fall–nonfall classification accuracy were obtained when calculation was performed for *C*4 rather than for each measurement condition. Therefore, it is a potential tool for assessing the risk of falls by measuring the COP of the elderly.

## Figures and Tables

**Figure 1:** Illustration of EMD decomposition of COP signal. (a–g) are original COP*x* signals, and corresponding EMD decomposition is from IMF1 to IMF6. *X*-axis is points index. Signal length is 30 seconds.

**Figure 2:** Experimental flowchart.

**Figure 3:** Decision tree classification results for *C*4 and the other four measurement conditions. Unit of *y*-axis is average testing group accuracy.

**Table 1:** Subject's personal information.

	Nonfall	Fall
Subject number	47	29
Gender (female/male)	F33/M14	F27/M2
Age (mean/std.)	71.72 (6.55)	70.65 (6.39)
BMI (mean/std.)	25.44 (2.91)	25.65 (2.94)

**Table 2:** Feature parameters and their code numbers.

Level	Symbol	Explanation
1	*x*, y	*x* = cop*x*; *y* = cop*y*
2	0, 1, 2, 3, 4, 5, 6	Raw signal = 0; IMF1 signal = 1; IMF2 signal = 2,…, IMF6 signal = 6
3	1, 2, 3, 4, 5	RMSD = 1; median frequency = 2; total frequency power = 3; approximate entropy = 4; sample entropy = 5

**Table 3:** Group statistics for *C*4 feature parameters between fall and nonfall groups. Data is represented as mean (standard derivation).

Features name	Fall	Nonfall	*p* value	<0.05^*∗*^; <0.01^*∗∗*^; <0.001^*∗∗∗*^
*x*.1.4	0.45 (1.12)	0.47 (0.11)	0.0011	^*∗∗*^
*x*.2.4	0.24 (0.06)	0.25 (0.06)	0.00061	^*∗∗∗*^
*x*.3.4	0.10 (0.03)	0.11 (0.03)	5.9E-0.5	
*x*.4.4	0.05 (0.01)	0.05 (0.01)	0.00014	^*∗∗∗*^
*x*.5.4	0.02 (0.007)	0.02 (0.007)	0.00824	^*∗∗*^
*y*.0.4	0.08 (0.03)	0.08 (0.03)	0.015	^*∗*^
*y*.2.4	0.23 (0.07)	0.24 (0.07)	0.01096	^*∗*^
*y*.4.4	0.05 (0.01)	0.05 (0.01)	0.02956	^*∗*^
*y*.5.4	0.02 (0.007)	0.02 (0.007)	0.00522	^*∗∗*^
*y*.6.4	0.01 (0.004)	0.01 (0.004)	0.04756	^*∗*^
*x*.0.5	0.54 (0.09)	0.55 (0.08)	0.0085	^*∗∗*^
*x*.1.5	0.34 (0.13)	0.36 (0.13)	0.00447	^*∗∗*^
*x*.2.5	0.19 (0.06)	0.20 (0.05)	0.00142	^*∗∗*^
*x*.3.5	0.10 (0.02)	0.10 (0.03)	5.10E-05	^*∗∗∗*^
*x*.4.5	0.05 (0.01)	0.06 (0.01)	7.24E-05	^*∗∗∗*^
*x*.5.5	0.02 (0.007)	0.02 (0.007)	0.015035	^*∗*^
*y*.0.5	0.41 (0.12)	0.45 (0.12)	1.70E-05	^*∗∗∗*^
*y*.1.5	0.32 (0.18)	0.34 (0.17)	0.04	^*∗*^
*y*.2.5	0.16 (0.06)	0.17 (0.07)	0.01	^*∗*^
*y*.4.5	0.05 (0.01)	0.05 (0.01)	0.03	^*∗*^
*y*.5.5	0.02 (0.004)	0.02 (0.007)	0.00439	^*∗∗*^
*y*.6.5	0.01 (0.004)	0.01 (0.004)	0.03607	^*∗*^
*x*.1.2	1.85 (0.8)	2.01 (0.82)	0.005982	^*∗∗*^
*x*.2.2	0.87 (0.20)	0.91 (0.21)	0.00594	^*∗∗*^
*x*.3.2	0.46 (0.10)	0.49 (0.11)	0.00594	^*∗∗*^
*x*.4.2	0.25 (0.05)	0.26 (0.05)	0.00594	^*∗∗*^
*x*.5.2	0.13 (0.03)	0.13 (0.05)	0.03749	^*∗*^
*y*.2.2	0.84 (0.22)	0.88 (0.24)	0.01992	^*∗*^
*y*.4.2	0.26 (0.06)	0.27 (0.06)	0.03622	^*∗*^
*y*.5.2	0.14 (0.03)	0.14 (0.03)	0.03622	^*∗*^

**Table 4:** Single feature with significant difference between fall and nonfall groups under different COP measurement conditions. Solid square means the *p* value is smaller than 0.05.

Feature	*C*4	OF	CF	CR	OR
*x*.2.1	■	■			■
*x*.3.1				■	■
*x*.4.1					■
*x*.5.1					■
*x*.6.1					■
*y*.5.1	■	■			
*y*.6.1	■	■			
*x*.1.2	■				
*x*.2.2	■				■
*x*.3.2	■		■	■	■
*x*.4.2	■			■	■
*x*.5.2	■				■
*y*.2.2	■			■	
*y*.4.2	■	■			
*y*.5.2	■	■			
*x*.2.3					■
*x*.3.3				■	■
*x*.4.3					■
*x*.5.3					■
*x*.6.3					■
*y*.5.3	■	■			
*y*.6.3	■	■			
*x*.1.4	■			■	■
*x*.2.4	■	■			■
*x*.3.4	■			■	■
*x*.4.4	■	■		■	■
*y*.5.4	■	■			■
*y*.0.4	■				
*y*.1.4				■	
*y*.2.4	■			■	
*y*.3.4			■		
*y*.4.4	■				
*y*.5.4	■				■
*y*.6.4	■				
*x*.0.5	■			■	■
*x*.1.5	■			■	■
*x*.2.5	■				
*x*.3.5	■			■	■
*x*.4.5	■			■	■
*x*.5.5	■				■
*y*.0.5	■		■	■	■
*y*.1.5	■			■	
*y*.2.5	■		■	■	
*y*.4.5	■				
*y*.5.5	■	■			■
*y*.6.5	■				

**Table 5:** Numbers of statistically significant features on different COP measurement conditions.

Measurement conditions	*C*4	OF	CF	CR	OR
All	35	11	4	17	27
Raw	3	0	1	2	2
EMD derived	32	11	3	15	25
IMF1	4	0	0	4	2
IMF2	7	2	1	3	4
IMF3	3	0	1	5	5
IMF4	6	2	0	3	5
IMF5	8	5	0	0	7
IMF6	4	2	1	0	2
Time domain (RMSD)	3	3	0	1	5
Frequency domain	10	4	1	4	9
Nonlinear domain	22	4	3	12	13

## Data Availability

The data were taken from a public database.

## Appendix

### A. COP Feature Distributions

Feature parameters and codes for enrollees can be accessed through the following link: https://github.com/loveso1G/C02E-1.git.

### B. Decision Tree Classification Resultsel

Results of classification with a decision tree for all features can be accessed through the following link: https://github.com/loveso1G/C02-2.git.
